# Morphological Variations of the Posterior Superior Iliac Spine in Chinese Population: Potential Effects on the Reliability of Palpation

**DOI:** 10.1155/2022/6290133

**Published:** 2022-08-08

**Authors:** Ji Qi, Jing Li, Haizhou Wang, Ruiyue Ping, Yikai Li, Haiyun Chen, Jiheng Zhan, Ping Chen, Bing Yang, Xiubing Yu, Qing Zhang, Dingkun Lin

**Affiliations:** ^1^Department of Orthopaedics, Guangdong Provincial Hospital of Traditional Chinese Medicine, Guangzhou 510120, China; ^2^Wang Jing Hospital, China Academy of Chinese Medical Sciences, Beijing 100102, China; ^3^The Second Clinical College, Guangzhou University of Chinese Medicine, Guangzhou 510120, China; ^4^Postdoctoral Research Station, Guangdong Provincial Hospital of Traditional Chinese Medicine, Guangzhou 510120, China; ^5^Department of Dermatology, Guangdong Provincial Hospital of Traditional Chinese Medicine, Guangzhou 510120, China; ^6^Southern Medical University, Guangzhou 510105, China

## Abstract

**Objectives:**

The posterior superior iliac spine (PSIS) is an important anatomical landmark often involved in spinal manipulation and surgical bone harvest. Hence, knowledge of variations in the PSIS may be predictive and valuable in clinical settings. Taking the complex morphology into account, the study is aimed at proposing a classification of PSIS in the Chinese population.

**Methods:**

An anatomical study was undertaken on 288 human ilia. First, the morphological features of variations in the PSIS were noted following visual inspection. Then, 12 variable anatomical parameters were measured in order to determine the differences based on morphology, side, and sex.

**Results:**

Overall, four types of PSIS were found among 288 bones, including type I “V-shape” (106, 36.8%), type II “U-shape” (121, 42.0%), type III “W-shape” (36, 12.5%), and type IV “ossification-shape” (25, 8.7%). There were no significant sex or bilateral differences in the morphological distribution of the PSIS (*p* > 0.05). Furthermore, the measurements showed that type I was the narrowest and type III the broadest (*p* < 0.05). Moreover, female specimens had an overall larger distance and width of surrounding landmarks (*p* < 0.05), and a significant difference was found in the width of the PSIS between the left and right sides (*p* < 0.05).

**Conclusion:**

The PSIS samples displayed multiple morphological variations and could be classified into four types. In addition, sex-based or bilateral differences existed in the size and relative positions. It is thus likely that differences in the morphology and asymmetry of the PSIS provide references for palpation, bone harvest, and other clinical settings.

## 1. Introduction

The posterior superior iliac spine (PSIS) is an important anatomical landmark behind the ilium, and it can be palpated from the body surface [1, 2]. Multiple clinical implications of the PSIS have been reported. First, the PSIS is the common site of bone marrow aspiration. Compared to the anterior superior iliac spine (ASIS), the greater area of the PSIS is able to provide larger samples with less pain [3]. Second, as a potential area for source tissue for a bone graft, the harder bone harvested from the PSIS is more suitable for intraoperative bone grafting. For these reasons, it can not only guarantee the efficacy but also reduce the cost of an allograft. In the clinic, the available cortical cancellous bone graft from this site can be used for the treatment of old fractures, bone defects, nonunion, joint replacement, revisions, and other surgeries [4–6]. Third, palpation of the PSIS during physical examination is an important method of identifying pelvic torsion and sacroiliac joint (SIJ) disorder [7]. Diagnosing SIJ disorder is difficult, because the main complaint is similar to back pain caused by other psychological factors, but injections of the PSIS to control analgesia are the most important diagnostic tool [8]. Furthermore, when using botulinum toxin to treat psoas spasm [9] or during the free-handed placement of a second sacral vertebra sacroiliac screw [10], the PSIS is the most ideal landmark. Thus, knowledge of PSIS morphology is helpful during a variety of clinical applications.

Adult skeletal morphology of the ilium is useful in forensic anthropology. First, an estimation of age using the iliac crest is a key component in establishing a biological profile [7, 11]. Second, owing to the great differences in anatomical morphology, sex can be distinguished by differing morphology. Specifically, there are significant differences in the morphological characteristics of the iliac crest, SIJ, auricular surface, and pubic symphysis between male and female [12–15]. Whether a difference in PSIS morphology exists between men and women is still unknown.

Since palpation of the PSIS may be affected by body position, its reliability is controversial [16]. Moreover, the PSIS is large in size and irregular in shape. To date, little is known about its anatomical morphology. Therefore, this anatomical study was carried out to determine the morphology of the PSIS, to supplement anatomy research of the ilium and provide an anatomical basis and data reference for surgery.

## 2. Materials and Methods

### 2.1. Ethics Statement

All procedures performed in this study involving human specimens were following the Declaration of Helsinki (as revised in 2013). The procedures were approved by the Ethics Committee of Guangdong Provincial Hospital of Chinese Medicine (No. ZM2021-128).

### 2.2. Specimen Collection

Except for malformations, fracture, and hypoplasia, a total of 288 intact dry Chinese ilia bones were collected from the Department of Anatomy, Southern Medical University.

### 2.3. Data Collection

The sex of each bone was determined according to the angle between the symphyseal surface margin and the inferior pubic ramus, as previously reported (Figure 1) [17]. All bones were observed and measured in order. First, the PSIS was classified based on its overall shape and size during visual inspection. Then, the anatomical structure was measured according to standard definitions and procedures. Twelve separate parameters were measured by the same observer using a digital calliper (DEGUQMNT MNT-200, Shanghai, China, accurate to 0.01 mm) and recorded in millimetres (Figure 2). The investigator had a 5-year experience of anatomical studies. To avoid intrainvestigator errors, each parameter was measured five times, and the mean of all datasets was then used to decrease the probability of errors. Each bone was measured as follows:

1. *L*_ab_: the distance between the PSIS (a) and the ASIS (b)
2. *L*_cd_: the distance between the ischial tuberosity (IT) (c) and the highest point of the iliac crest (HIC) (d)
3. *L*_ac_: the distance between the PSIS (a) and IT (c)
4. *L*_ae_: the distance between the PSIS (a) and the pubic tuberosity (PT) (e)
5. *L*_af_: the distance between the PSIS (a) and the midpoint of the posterior edge of the auricular surface (AS) (f)
6. *L*_0_: the distance between the tip and the widest part of the PSIS
7. *L*_ag_: the distance between the PSIS (a) and the transition of the iliac crest (TIC) (g)
8. *W*_0_: the tip width of the PSIS
9. *W*_max_: the maximum width of the PSIS
10. *W*_0_/*W*_max_: the ratio of *W*_0_ to *W*_max_
11. *W*_g_: the width of the TIC
12. *T*_0_: the tip thickness of the PSIS

### 2.4. Statistical Analysis

Numerical data were presented as mean and standard deviation (SD), and categorical data were presented as number and frequency. Normal distribution within each group was tested with the *Kolmogorov-Smirnov* test. Differences in sex and side distribution of PSIS morphological classifications were tested using the chi-square test. The differences in anatomical parameters based on sex and side were evaluated by independent sample *t*-test. Differences in the anatomical parameters among morphological classifications were analyzed by one-way ANOVA. A two-side *p* value < 0.05 was considered statistically significant. All statistical analyses were performed by IBM SPSS 23.0 software (SPSS Inc., Chicago, IL, USA).

## 3. Results and Discussion

### 3.1. Morphological Classification of the PSIS

Among 288 human ilia, four types of PSIS morphology were found (Figures 3 and 4). Type I (V-shape, 36.8%) and type II (U-shape, 42.0%) were more common. The frequency of type III (W-shape) and type IV (ossification-shape) was 12.5% and 8.7%, respectively.

### 3.2. Morphological Differences in Measurements

As shown in Table 1, differences existed in anatomical parameters among the four morphological types, except for *W*_g_ and *L*_0_ (*L*_ab_, *F* = 4.455, *p* = 0.004; *L*_cd_, *F* = 3.360, *p* = 0.019; *L*_ac_, *F* = 5.252, *p* = 0.002; *L*_ae_, *F* = 2.739, *p* = 0.044; *L*_af_, *F* = 3.983, *p* = 0.008; *L*_ag_, *F* = 4.668, *p* = 0.009; *W*_0_, *F* = 97.072, *p* < 0.001; *W*_max_, *F* = 2.774, *p* = 0.042; *W*_0_/*W*_max_, *F* = 75.91, *p* < 0.001; *L*_0_, *F* = 1.866, *p* = 0.136; *T*_0_, *F* = 33.168, *p* < 0.001).

For *L*_ab_, type I was shorter than type III (*p* = 0.006) and type IV (*p* = 0.004). For *L*_cd_, type I was shorter than type IV (*p* = 0.008). For *L*_ac_, type I was shorter than type II (*p* < 0.001), type III (*p* = 0.017), and type IV (*p* = 0.022). For *L*_ae_, type I was shorter than type II (*p* = 0.005). For *L*_af_, type I was shorter than type II (*p* = 0.001) and type III (*p* = 0.038). For *L*_ag_, type I was shorter than type III (*p* = 0.009) and type IV (*p* = 0.004), and type II was shorter than type III (*p* = 0.020) and type IV (*p* = 0.009). For *W*_0_, type I was the smallest, compared to type II (*p* < 0.001), type III (*p* < 0.001), and type IV (*p* < 0.001). For *W*_max_, type I was shorter than type III (*p* = 0.013), while type II was shorter than type III (*p* = 0.007). For *W*_0_/*W*_max_, type I was the smallest, compared to type II (*p* < 0.001), type III (*p* < 0.001), and type IV (*p* < 0.001), while type II was shorter than type IV (*p* < 0.001), and type III was greater than type IV (*p* < 0.001). For *L*_0_, type I was greater than type IV (*p* = 0.027). For *T*_0_, type I was the smallest compared to type II (*p* < 0.001), type III (*p* < 0.001), and type IV (*p* < 0.001), while type II was greater than type IV (*p* = 0.035).

### 3.3. Sexual Difference

No significant sexual difference was found in the morphological distribution of the PSIS in both bone specimens (*p* > 0.05), as shown in Table 2. However, the sexual difference in anatomical parameters was significant, as shown in Table 3. For *L*_ab_, *L*_cd_, *L*_ac_, *L*_ag_, and *T*_0_, female specimens had greater measurements than males (*L*_ab_, 151.80 ± 9.98 mm in females vs. 148.30 ± 9.31 mm in males, *p* = 0.004; *L*_cd_, 204.73 ± 13.12 mm in females vs. 197.27 ± 12.38 mm in males, *p* < 0.001; *L*_ac_, 149.20 ± 10.15 mm in females vs. 146.40 ± 9.15 mm in males, *p* = 0.018; *L*_ag_, 74.03 ± 11.10 mm in females vs. 71.13 ± 9.79 mm in males, *p* = 0.029; *T*_0_, 8.55 ± 5.10 mm in females vs. 7.30 ± 4.32 mm in males, *p* = 0.029). No difference was found in the other seven parameters (*p* > 0.05).

### 3.4. Bilateral Difference

There was no significant bilateral difference in the morphology of PSIS in bone specimens (Table 2; *p* > 0.05). However, it was evident that a bilateral difference existed in a certain anatomical parameter, as shown in Table 3. For *W*_0_ and *W*_0_/*W*_max_, the right sides were greater than the left ones (*W*_0_, 8.05 ± 3.18 mm in right vs. 7.16 ± 3.13 mm in left, *p* = 0.017; *W*_0_/*W*_max_, 0.45 ± 0.19 in right vs. 0.40 ± 0.17 in left, *p* = 0.007). No significant difference was found in the other 10 parameters (*p* > 0.05).

## 4. Discussion

### 4.1. PSIS Morphological Variation and Its Relationship to Body Size

Although the morphology of the hip bone is important in orthopaedics, chiropractic, and even in medicolegal expertise, the morphology and variation of the PSIS are rarely reported. In this study, the morphology of the PSIS from 288 bone specimens was summarized and measured, and the results revealed that variation in PSIS morphology is not rare. In terms of general morphology, PSISs could be classified into type I (V-shape), type II (U-shape), type III (W-shape), and type IV (ossification-shape). The four morphological types of the PSIS varied in sharpness, width, and thickness. Among the types, type II (42.0%) was the most common, followed by types I (36.8%) and III (12.5%), with type IV (8.7%) being the least common.

Despite of the difficulty to estimate the accurate body size, we still identified the overall size of these hip bones in this study. *L*_ab_ and *L*_cd_ were measured, to give average lengths of 150.59 mm and 202.14 mm. In related studies, Glinski et al. measured the *L*_ab_ distance on 11 hip bones as 164.77 ± 3.63 mm [18]; and Okamoto et al. noted *L*_cd_ distances of 21.2 ± 0.8 cm for men and 19.8 ± 0.9 cm for women [19]. Compared to the reported anatomical data, the shorter distances in this study may be attributed to the sample size and ethnic differences. Despite this, we found that PSIS morphology seemed to be related to the overall size of the hip bone. Among the 288 specimens, type I had shorter lengths of *L*_ab_ and *L*_cd_ in comparison with types III and IV, possibly indicating that V-shape PSISs are common in small-sized hip bones. Taking the relationship between iliac and human body size into consideration, the results demonstrated that a thin population may be more likely to have a V-shape PSIS. From this view, owing to the sharp shape and the lower amount of subcutaneous tissue, the PSIS could be easily palpated during a physical test easily in the thin population, which is consistent with clinical experience.

### 4.2. Potential Effects of PSIS Morphometrical Differences on Clinical Applications

Except for the overall size, this study found that the main variations in the PSIS existed in the topical anatomical parameters. There were multiple significant differences in the measurements of the landmarks among the four morphological types. At the tip of the PSIS, *W*_0_ and *T*_0_ reflected the width and thickness separately, and results showed that both *W*_0_ and *T*_0_ of type I were significantly shorter than for the other three types. The measurements demonstrated that the posterior tip of V-shape PSIS was narrower and thinner, showing similar characteristics to the general morphology. From the tip to the iliac crest, the PSIS gradually became wider in morphology. *W*_max_, *W*_0_/*W*_max_, the distance of *L*_0_, and *L*_ag_ reflected the maximum width surrounding the PSIS, the width trend, the longest distance from the posterior tip to the widest part, and the posterior length of the iliac crest, separately. *W*_max_ and *L*_ag_ of type III were longer than type I and type II; however, type I had the lowest width ratio (*W*_0_/*W*_max_) and the longest *L*_0_ compared with the other three types. The difference may not only reveal the wider variation of the W-shape but also demonstrate the sharper variation of the V-shape in PSIS morphology. These types of morphological differences have been neglected in previous studies. In terms of the result, it is reasonable to assume that the sharper V-shape PSIS or the obtuse W-shape PSIS is very different when palpated. Furthermore, the wider PSIS in types II and III may be more suitable for bone marrow aspiration and larger graft harvest.

Ossification-shape PSIS was another specific variation found in this anatomical study. The most obvious variation in the morphology was the irregular presence of bone ossification. Visually, the ossification clearly highlighted the iliac crest as well as their size and location are different; however, the location and size of the bone ossification were diverse. The effect of the morphological variation on the accuracy of the palpated sites seems to be a trouble during the physical test. Therefore, this type requires greater attention in the clinical setting, since the occurrence rate was 8.7% in this study and the morphology may influence the accuracy of palpation and positioning. Few previous studies have focused on this point. Multiple tendons and ligaments attach around the PSIS, including the sacrotuberous ligament, long posterior sacroiliac ligament, erector spinae, and multifidus muscles. The roles of the above ligaments and tendons in restricting sacral movement and assisting with pelvic stabilization have been derived from a previous study [20]. Along with increasing age, continuous mechanical traction on the insertion sites of tendons and ligaments is one of the common reasons for the development of ossification. Thus, we suggest that the ossification in this region corresponded to bony proliferation frequently encountered in individuals of middle-age and the elderly. In addition to age, degeneration and ankylosing spondylitis may promote bony proliferations. In the future, the correlation between the presence of the ossification-shape type and disease remains to be investigated.

SIJ injection is one kind of useful therapy when treating SIJ pain or disorder. Accurate placement of the injection is essential for achieving a satisfying result. The PSIS is a reference landmark during the procedure, and *L*_af_ is of vital importance for ensuring the location of the SIJ and puncture depth. The result of this study found the mean distance was 16.32 mm, which is similar to result found in published literature (16.8 mm) [21]. Furthermore, the distance was different among the four types, as type I was shorter than in types II and III. That is, if a V-shape PSIS was found during palpation or radiological test, the SIJ would be closer to the PSIS. Under this condition, it would be preferable to make a related superficial puncture during the SIJ injection, and the puncturing depth should be controlled.

Multiple landmarks of the pelvic skeleton can be palpated superficially, such as the PSIS, HIC, IT, PT, and ASIS. During the process of PSIS palpation, the relative distance to other landmarks could provide reference during superficial location. In this study, we also found that the *L*_ae_ of type I was lower than type II, while the *L*_ac_ of type I was lower than in other three types. That is, if a shorter distance from PSIS to PT or to IT was found, the PSIS would likely to be V-shape (95% confidence interval: *L*_ac_, 143.46-147.07 mm; *L*_ae_, 152.41-156.32 mm). Thus, all measurements may be helpful for PSIS identification during clinical palpation.

### 4.3. Sexual and Bilateral Differences in PSIS Morphology and Morphometry

Owing to the incomplete records of skeletons during their conservation, the sex of the specimens was not previously determined. Thus, sex determination based on bone measurement was applied according to the above reported method. Based on this, the sexual difference in the PSIS was evaluated, except for morphological variation. Although no difference in morphological distribution was found between the male and the female skeletons, the measurements of landmarks remained different. Firstly, the length of *L*_ab_, *L*_cd_, and *L*_ag_ of the male was shorter than for the female, possibly indicating that the larger female iliac bone is associated with the anatomy and physical performance of the female pelvis. Secondly, for the topical variation in the PSIS, only *T*_0_ of the male was thinner than in the female. This result suggested that female PSIS may be more difficult to be palpated superficially, but could provide a greater harvest of bone during surgery.

Moreover, this study found a potential difference in the anatomy of the bilateral hip bones. In previous studies, iliac crest asymmetry has been considered as a common phenomenon noted during radiology [22]. However, it remains unknown whether a difference of asymmetry exists in the PSIS. In the current study, we found that morphological distributions on the right side were similar to those on the left side; meanwhile, the width of *W*_0_ and the ratio of *W*_0_/*W*_max_ on the left side were less than the right side. During the diagnosis of SIJ disorder, asymmetry of the PSIS is commonly considered as a key physical sign. Furthermore, in the treatment of SIJ disorder, if a postoperative symmetrical landmark of the PSIS is achieved following spinal manipulation, the treatment would be considered successful. Despite the 288 hip bones measured in this study not all being paired, asymmetrical widths of PSISs may exist in healthy individuals. If so, the physical asymmetry might be a bias in the accuracy of palpating and positioning, especially in the diagnosis of SIJ diseases.

However, limitations still exist in this study. Firstly, the imbalance in the sex of the bones may have affected the analysis of sex distribution. Secondly, the uneven and irregular surface of the PSIS may result in unpredictable errors during measurement. Furthermore, owing to objective problems such as the limited number of dried bone specimens and the difficulty of storage, the specimens measured in this study were not completely paired and therefore cannot yet reflect the problem of left-right asymmetry in an individual. In addition, because of incomplete previous records, it was at times difficult to give an accurate age of a bone. Thus, both the age-related morphological variation and presence of ossification were still unclear. Therefore, a more detailed analysis based on three-dimensional reconstruction remains to be performed in the future, which will provide a digital platform for the study and help to clarify for the shortcomings of the current study.

## 5. Conclusions

In summary, the present study found that there were four morphological types of the PSIS: type I (V-shape), type II (U-shape), type III (W-shape), and type IV (ossification-shape). U-shape PSIS was greatest in number, and no sexual or side-related difference was found in the morphology of the PSIS. The V-shape PSIS was the narrowest, and the W-shape PSIS was the broadest. The V-shape PSIS was often found on small-sized hip bones, which might be common in a thin population and be easily palpated. In addition, the morphology of ossification was often irregular, and certain sexual differences or asymmetry may exist in the topical parameters of the PSIS. Furthermore, female specimens had an overall larger length and width of surrounding landmarks, and an asymmetrical difference existed in the width of the PSIS. All these variations may need to be considered during clinical procedures such as palpation, positioning, puncture, and injection.

## Figures and Tables

**Figure 1:** Distinguishing sex according to the angle between the symphyseal surface margin and inferior pubic ramus. (a) Male specimen with the angle > 137°; (b) female specimen with the angle < 137°.

**Figure 2:** Measurement of anatomical parameters.

**Figure 3:** Sketches of different types of posterior superior iliac spine are shown on the diagram. (a) Type I: V shape; (b) type II: U-shape; (c) type III: W-shape; (d) type IV: ossification-shape.

**Figure 4:** Specimens of different types of posterior superior iliac spine. (a, e) Type I: V-shape; (b, f) type II: U-shape; (c, g) type III: W-shape; (d, h) type IV: ossification-shape.

**Table 1:** Difference in anatomical parameters of the posterior superior iliac spine (mean ± SD).

	Classification				*F*	*p*
	Type I (*n* = 106)	Type II (*n* = 121)	Type III (*n* = 36)	Type IV (*n* = 25)		
*L*_ab_ (mm)	148.33 ± 9.36^b,c^	150.86 ± 10.16	153.53 ± 8.10	154.58 ± 10.95	4.455	0.004^∗^
*L*_cd_ (mm)	199.37 ± 13.74^b,c^	202.73 ± 12.83	204.81 ± 12.06	207.19 ± 13.84	3.360	0.019^∗^
*L*_ac_ (mm)	145.27 ± 9.39^a,b,c^	149.97 ± 10.00	149.73 ± 9.64	150.21 ± 9.26	5.252	0.002^∗^
*L*_ae_ (mm)	154.36 ± 10.13^a^	158.10 ± 9.65	156.76 ± 10.73	156.72 ± 8.13	2.739	0.044^∗^
*L*_af_ (mm)	15.10 ± 4.72^a,b^	17.24 ± 4.83	17.06 ± 4.33	15.98 ± 6.10	3.983	0.008^∗^
*W*_g_ (mm)	11.71 ± 3.62	11.28 ± 1.98	11.57 ± 2.28	12.28 ± 1.61	1.119	0.342
*L*_ag_ (mm)	71.48 ± 10.43^b,c^	72.16 ± 11.63^b,c^	76.84 ± 8.04	78.27 ± 8.15	4.668	0.003^∗^
*W*_0_ (mm)	4.77 ± 2.04^a,b,c^	9.28 ± 2.28	10.38 ± 2.27	7.34 ± 2.83	97.072	<0.001^∗^
*W*_max_ (mm)	17.97 ± 2.88^b^	17.88 ± 2.73^b^	19.34 ± 3.35	18.57 ± 2.59	2.774	0.042^∗^
*W*_0_/*W*_max_	0.27 ± 0.13^a,b,c^	0.53 ± 0.14^c^	0.55 ± 0.15^c^	0.40 ± 0.13	75.91	<0.001^∗^
*L*_0_ (mm)	23.89 ± 8.63^c^	22.49 ± 6.48	22.35 ± 8.24	20.17 ± 5.99	1.866	0.136
*T*_0_ (mm)	4.99 ± 2.96^a,b,c^	10.52 ± 4.90^c^	8.96 ± 4.52	8.56 ± 4.70	33.168	<0.001^∗^

Note: ^∗^*p* < 0.05; ^a^*p* < 0.05 vs. type II; ^b^*p* < 0.05 vs. type III; ^c^*p* < 0.05 vs. type IV.

**Table 2:** Gender or side related morphological distribution of PSIS (*n*, %).

Variable		Classification				Total
		Type I	Type II	Type III	Type IV	
Gender^∗^	Female	66 (35.1)	78 (41.5)	23 (12.2)	21 (11.2)	188 (100.0)
	Male	40 (40.0)	43 (43.0)	13 (13.0)	4 (4.0)	100 (100.0)
Side^#^	Left	56 (38.1)	63 (42.9)	14 (9.5)	14 (9.5)	147 (100.0)
	Right	50 (35.5)	58 (41.1)	22 (15.6)	11 (7.8)	141 (100.0)

Note: ^∗^gender difference, *χ*^2^ = 4.357, *p* = 0.225 > 0.05; ^#^bilateral difference, *χ*^2^ = 2.560, *p* = 0.465 > 0.05.

**Table 3:** Gender or bilateral differences in anatomical parameters around PSIS (mean ± SD).

Parameter	Gender				Side			
	Male (*n* = 100)	Female (*n* = 188)	*t*	*p*	Left (*n* = 147)	Right (*n* = 141)	*t*	*p*
*L*_ab_ (mm)	148.30 ± 9.31	151.80 ± 9.98	2.897	0.004^∗^	150.66 ± 9.11	150.50 ± 10.66	0.136	0.892
*L*_cd_ (mm)	197.27 ± 12.38	204.73 ± 13.12	4.679	<0.001^∗^	201.42 ± 12.02	202.89 ± 14.58	-0.937	0.349
*L*_ac_ (mm)	146.40 ± 9.15	149.20 ± 10.15	2.380	0.018^∗^	148.31 ± 9.84	148.14 ± 9.97	0.153	0.878
*L*_ae_ (mm)	156.72 ± 9.14	156.29 ± 10.37	-0.349	0.727	156.86 ± 9.82	156.00 ± 10.09	0.733	0.464
*L*_af_ (mm)	15.10 ± 4.76	16.97 ± 4.91	3.114	0.192	16.12 ± 5.11	16.53 ± 4.75	-0.700	0.485
*W*_g_ (mm)	11.28 ± 2.85	11.72 ± 2.64	1.307	0.192	11.57 ± 2.62	11.57 ± 2.82	-0.005	0.996
*L*_ag_ (mm)	71.13 ± 9.79	74.03 ± 11.10	2.193	0.029^∗^	73.49 ± 11.19	72.54 ± 10.26	0.751	0.453
*W*_0_ (mm)	7.36 ± 3.25	7.71 ± 3.15	0.893	0.372	7.16 ± 3.13	8.05 ± 3.18	-2.391	0.017^∗^
*W*_max_ (mm)	18.08 ± 2.72	18.20 ± 2.98	0.337	0.736	18.24 ± 2.82	18.06 ± 2.96	0.522	0.602
*W*_0_/*W*_max_	0.41 ± 0.19	0.43 ± 0.18	0.874	0.383	0.40 ± 0.17	0.45 ± 0.19	-2.709	0.007^∗^
*L*_0_ (mm)	22.44 ± 6.80	22.97 ± 7.95	0.569	0.570	23.10 ± 6.33	22.46 ± 8.67	0.715	0.475
*T*_0_ (mm)	7.30 ± 4.32	8.55 ± 5.10	2.198	0.029^∗^	8.47 ± 5.41	7.76 ± 4.23	1.245	0.214

Note: ^∗^*p* < 0.05.

## Data Availability

The data used to support the findings of this study are available from the corresponding author (Dingkun Lin) upon request.
